The article "Circular RNA CircITGA7 Promotes Tumorigenesis of Osteosarcoma via miR-370/PIM1 Axis" was retracted in 2023. Reasons: unreliable results or conclusions; concerns about the data; concerns about the peer review; concerns about the citations.

# Circular RNA CircITGA7 Promotes Tumorigenesis of Osteosarcoma via miR-370/PIM1 Axis

**DOI:** 10.1155/2020/1367576

**Published:** 2020-09-10

**Authors:** Chuanwu Fang, Xiaohong Wang, Dongliang Guo, Run Fang, Ting Zhu

**Affiliations:** ^1^Department of Orthopedic Surgery, The Third Affiliated Hospital of Anhui Medical University, Hefei, Anhui, China; ^2^Department of Oncology, The Third Affiliated Hospital of Anhui Medical University, 390 Huaihe Road, Hefei, Anhui, China

## Abstract

Many studies have shown that there are many circular RNA (circRNA) expression abnormalities in osteosarcoma (OS), and this abnormality is related to the development of osteosarcoma. But at present, it is unclear as to what circITGA7 has in the OS and what it does. In this study, qRT-PCR was used to detect the expression of circITGA7, miR-370, and PIM1 mRNA in OS tissues and cells. The CCK-8 assay was used to detect the effect of circITGA7 on cell proliferation. Later, the transwell assay was used to detect cell migration and invasion. The dual-luciferase reporter assay confirmed the existence of the targeting relationship between circITGA7 and miR-370, and miR-370 and PIM1. We found that circITGA7 was upregulated in OS tissues and cell lines. Knockdown of circITGA7 weakened the cell's ability to proliferate and metastasize. Furthermore, we observed that miR-370 was negatively regulated by circITGA7, while PIM1 was positively regulated by it. A functional assay validated that circITGA7 promoted OS progression via suppressing miR-370 and miR-370 affected OS proliferation and migration via PIM6 in OS. In summary, this study shows that circITGA7 promotes OS proliferation and metastasis via miR-370/PIM1.

## 1. Background

Osteosarcoma (OS) is a malignant cancer with a worldwide incidence of 0.2% [1]. It is, nevertheless, one of the subjects of huge interest to surgeons. One of the characteristics of osteosarcoma is that it tends to occur in adolescents, representing a bimodal pattern [2]. At the same time, osteosarcomas often occur in the distal femur or proximal tibia [3]. Because osteosarcomas do not have precancerous lesions or in situ cancers, when the diagnosis of osteosarcomas is made, the lesions that have occurred are often already malignant tumors [4]. It is, therefore, necessary to carry out the research of early diagnosis and explore the biomarker of early diagnosis and treatment [5].

Screening for molecular markers of cancer depends on whether there are differences in the molecular content between cancer cells and normal cells [6]. Alpha-fetoprotein, for example, is a glycoprotein found to be expressed at very low levels in the serum of normal adults, but high concentrations in cancer samples [7]. Similarly, some small molecules, such as circular RNA (circRNA), show differential expressions between cancer cells and normal cells. CircRNAs, usually produced in eukaryotic cells, participated in the regulation of various intracellular metabolisms in cells and have differential expression in various cancer cells [8]. For example, according to Wang and Li, circ_0067934 gene is highly expressed in human non-small-cell lung cancer (NSCLC). In in vitro experiments, the inhibition of the expression of this gene can significantly reduce the proliferation and invasion of NSCLC cells [9]. At the same time, due to the circular structure of circRNA, without free ports, it is not easy to be degraded by RNA exonuclease, so it has different stability and conservation compared to linear RNA in cells. Therefore, it is considered a promising biomarker for precision medicine of tumors [8].

One of a class of small molecules closely related to cell metabolism and process is miRNA [10]. miRNAs are involved in regulating gene expression in a variety of ways [11]. For example, miRNA competitively binds RNA-binding proteins, thereby blocking the inhibition of mRNA and RNA-binding proteins and thus regulating the expression of related genes [12]. In addition, certain miRNAs may be degraded when stimulated by specific stimulus factors, leading to the reactivation of related repressed mRNAs, thereby regulating the expression of related genes in response to the stimulus factors [11]. Similarly, miRNAs can act as oncogenes, or in some cases as tumor suppressors, to play a role in the progression of cancer [13]. Studies have found that miR-223 is shown to be upregulated in metastatic gastric cancer cells. Studies have shown that the transcription factor twist-stimulated miR-223 downregulates the expression of EPB41L3 after transcription by directly targeting its 3′-nontranslation regions, thus enhancing the migration and subsequent invasion ability of nonmetastatic gastric cancer cells as a regulatory factor [14].

CircITGA7 is a novel circular RNA, and ITGA7 is located on the human chromosome 12q13. Related studies have shown that circITGA7 is significantly dysregulated in a variety of human cancers, such as colorectal cancer and thyroid cancer. For example, previous studies have shown that circITGA7 is found to be significantly downregulated in colorectal cancer (CRC), inhibiting the proliferation and metastasis of CRC cells by inhibiting the Ras signaling pathway and promoting the transcription of ITGA7 [15]. At the same time, it is found that circITGA7 can also inhibit the proliferation of CRC by sponging miR-3187-3p and increasing the expression of ASXL1. Therefore, circ-ITGA7 may be a potential diagnostic biomarker and treatment target for CRC [16]. CircITGA7, upregulated in thyroid cancer cells, can directly bind to miR-198, reduce the inhibitory effect of miR-198 on the expression of target FGFR1, and regulate the metastasis and proliferation of TC cells, and it can be a potential marker for TC diagnosis or progression [17]. However, the role of circITGA7 in osteosarcomas is still unclear. Therefore, the focus of this research is to explore the potential functions of osteosarcomas.

In this study, the expression pattern of circITGA7 in osteosarcoma cells and the role of circITGA7 in promoting the proliferation, migration, and invasion of osteosarcoma cells were examined. The mechanism of circITGA7 in competitively binding miR-370 to regulate downstream target gene PIM1 was investigated. Our study demonstrates the potential of the circITGA7/miR-370/PIM1 axis as biomarkers for early screening, diagnosis, and monitoring of treatment progression for osteosarcoma.

## 2. Material and Methods

### 2.1. Human Tissue Samples

The osteosarcoma tissue and related normal tissues of 15 osteosarcoma patients from the Third Affiliated Hospital of Anhui Medical University were collected. The study period was between January 2010 and January 2018. Whole osteosarcoma samples were gathered from 15 OS patients and healthy controls. The patients had not received any prior chemotherapy, radiotherapy, or any other adjuvant treatment before surgery. The Research Ethics Committee of the Third Affiliated Hospital of Anhui Medical University approved this study, and all patients gave their written informed consent in this study.

### 2.2. Cell Lines and Cell Culture

The human OS cell lines (MG-63, HOS, U2OS, and SW1353) were procured from ATCC (Manassas, USA). The cells were cultured in a 37°C, 5% CO_2_ incubator using RPMI-1640 medium. 10% FBS (BI, Israel), 100 U/mL penicillin, and 100 *μ*g/mL streptomycin were used as supplements in the medium.

### 2.3. RNA Extraction and qRT-PCR

According to the manufacturer's instructions, total RNA was isolated from osteosarcoma tissue/cell line and related normal tissue/cell line using the TRIzol reagent. NanoDrop 2000c (Thermo Scientific, USA) was used for RNA quantification and quality examination. Using a SYBR Green PCR Kit (Vazyme, Nanjing, China), 2 *μ*g of total RNA was reverse-transcribed to cDNA. Subsequently, a qRT-PCR assay was conducted using QuantStudio™ 6 Flex (Thermo Fisher, USA) on an ABI 7500 according to the company's protocol. Primers involved in this study were designed and purchased from Sangon Biotech (Shanghai, China). U6 was used to normalize the mRNA expression of miR-370, and the mRNA expression of PIM1 was normalized to GAPDH.

### 2.4. Cell Counting Kit-8 Proliferation Assay

The cell proliferation assay was done according to the company's protocol of the CCK-8 kit (Dojindo Laboratories, Japan). In brief, nearly 1000 transfected cells in 100 *μ*L were grown in each well of 96-well plates. As indicated time points in the figure, cells in each well were treated with 10 *μ*L CCK-8 solution and subsequently incubated at 37°C for 2 hours. Then, a Varioskan Flash Multimode Reader MB-580 (HEALES, China) was employed to measure the optical density at 450 nm. Five replicates were used in each group of cells.

### 2.5. Transwell Migration and Invasion Assays

In this assay, transwell permeable supports were employed, with a polycarbonate membrane which was coated with Matrigel (Corning Inc., USA) (for invasion tests) or without Matrigel (for migration tests). 24 hours after transfection, the cells were seeded in the upper layer in 100 *μ*L serum-starved RPMI-1640, and then, 600 *μ*L of medium with 10% FBS was added to the bottom layer. After 48 hours of incubation, the cells on the top layer of the transwell chamber were wiped with cotton swabs, and methanol was used to fix the cells in the lower surface for 10 minutes, and subsequently, cells were stained with 10 *μ*g/mL of diamidino-2-phenylindole (DAPI) (Solarbio, Beijing, China) at room temperature for 15 minutes. A 200x fluorescence inverted microscope (Mshot, China) was used to photograph and count the stained cells in ten randomly selected fields.

### 2.6. Dual-Luciferase Reporter Assay

Approximately 5000 cells were seeded into each well of 96-well plates and subsequently cotransfected with associated plasmids and miRNA mimics or inhibitors. Lipofectamine 2000 was employed as a transfection reagent. After 48 hours of incubation, a dual-luciferase reporter assay (Promega, USA) was used to measure the luciferase activity. Independent tests were done in triplicate. For the normalizations of relative luciferase activity, it was renilla luciferase that was used as an internal control. siRNAs were designed and synthesized by RiboBio (Guangzhou, China) as follows: si-NC: 5′–UUCUCCGAACGUGUCACGUTT–3′; si-circITGA7: 5′-CCUAUAAUUGGAAGGACCUTT-3′. The plasmid was synthesized by RiboBio (Guangzhou, China).

### 2.7. Statistical Analysis

Results are shown as the mean ± SD. To measure the difference between two groups, Student's *t*-test was employed, and one-way ANOVA was used to assess differences between more than two groups. *P* < 0.05 was considered significant.

## 3. Results

### 3.1. CircITGA7 Was Upregulated in OS Tissues and Cell Lines

To investigate the functions of circITGA7 in osteosarcoma, at first, we studied its expression in osteosarcoma tissues and cell lines. Using qRT-PCR analysis, it was demonstrated that compared with normal tissues, the expression of circITGA7 in osteosarcoma tissue had increased significantly (Figure 1(a)). Moreover, the circITGA7 expression level was significantly elevated in two OS cell lines (U2OS and SW1353) compared to the normal human cell line hFOB 1.19. Therefore, these two cell lines were selected for subsequent research (Figure 1(b)). The discoveries implied that circITGA7 could play a carcinogenic role in OS.

### 3.2. CircITGA7 Facilitated OS Cell Proliferation, Migration, and Invasion In Vitro

To explore the impact of circITGA7 on the biological function of OS cells, we used siRNA (si-circITGA7) to silence the circITGA7 expression in U2OS cells and the circITGA7 level was reduced by 43 percent (Figure 1(c)). CCK-8 assays were used to measure its effect. It showed that knockdown of circITGA7 could attenuate the proliferation ability of the SW1353 and U2OS cells (Figures 1(d) and 1(e)). Transwell assays illustrated that the invasive and migratory capabilities of SW1353 and U2OS cells were attenuated by silencing circITGA7 (Figures 2(a)–2(d)).

### 3.3. CircITGA7 Could Upregulate the Expression of PIM1 by miR-370

It has been shown that circRNAs can function as competing RNAs to bind miRNAs in the cytoplasmic space. We assessed binding between circITGA7 and miRNAs using online bioinformatics databases (miRDB, miRTarbase, and miRmap). The miR-370 was shown to have binding sites for circITGA7 as demonstrated by software prediction methods, and the expression of miR-370 in OS cells SW1353 and U2OS increased by 2.5 times and 4 times after the knockdown of circITGA7, respectively (Figure 3(c)). In order to validate the interaction between miR-370 and circITGA7, wild-type (wt) or mutant (mut) targeted sites of miR-370 in circITGA7 were cloned into pGL3 plasmid. Findings obtained from the dual-luciferase reporter assay showed that miR-370 mimics considerably reduced the luciferase activity driven by wild-type circITGA7 in SW1353 and U2OS cells (Figures 3(a) and 3(b)). But the mutant circITGA7 was not impacted by miR-370. Furthermore, the binding site of miR-370 in 3′-UTR of PIM1 was obtained by analysis. We then examined the interaction between miR-370 and PIM1 by a dual-luciferase reporter assay (Figure 3(d)). PIM1 expression was evidently shown to be lower in SW1353 cells transfected with miR-370 than those cells with other processing groups (Figure 3(e)). Further investigation of PIM1 expression identified that anti-miR-370 could reverse the downregulation of PIM1 induced by circITGA7 knockdown in OS cells (Figure 3(f)). Taken as a whole, our results indicated that circITGA7 could upregulate PIM1 expression by miR-370.

### 3.4. miR-370 Reversed the Effect of CircITGA7

Using CCK-8 and transwell assay, we demonstrated that miR-370 acted as a tumor suppressor in OS. The results showed that miR-370 overexpression suppressed cell proliferation and migration in U2OS (Figures 4(a) and 4(c)); however, miR-370 knockdown enhanced cell proliferation and migration in SW1353 (Figures 4(b) and 4(d)).

In order to further explore the role of the circITGA7/miR-370 axis in OS, anti-miR-370 was arranged to be transfected into circITGA7 silenced SW1353 cells. CCK-8 and transwell assays were used to examine the effect of this treatment on OS cell proliferation and metastasis. Based on this, it was found that the proliferation and metastasis of SW1353 cells were inhibited due to downregulation of circITGA7 and that transfection with anti-miR-370 could partially reverse this inhibitory effect (Figures 4(e)–4(h)).

### 3.5. The Knockdown of PMI1 Partially Impeded the Effects of miR-370 Suppression on OS Cells

The above studies indicate that PIM1 is the target gene of miR-370. In order to continue to deeply investigate whether the effect of miR-370 on the physiological function of OS cells depends on PIM1 expression, we used siRNA (si-PIM1) to knock down PIM1 on OS cells that had been transfected with anti-miR-370 (Figures 4(i) and 4(j)). As shown in the figure, after knocking down PIM1, the cell proliferation and metastasis of SW1353 and U2OS were severely hindered. In conclusion, circITGA7 affected OS cell proliferation and migration through the miR-370/PIM1 axis.

## 4. Discussion

The results of our study showed that circITGA7 expression in osteosarcoma tissues or cells was significantly higher than that in corresponding normal tissues or cells. In in vitro experiments, si-circlTGA7 was used to knock down circITGA7 in SW1353 and U2OS cells. The results showed that circITGA7 knockdown reduced the proliferation of SW1353 and U2OS cells and dramatically checked the migration and invasion of osteosarcoma cells. To investigate the regulatory mechanism of circITGA7 in osteosarcoma, we found that circITGA7 promoted the progression of osteosarcoma cells by regulating the miR-370/PIM1 axis.

CircRNAs lack free 3′ or 5′ ends due to their circular structure, which makes it difficult for conventional mechanisms to degrade them. This structural characteristic results in a long half-life and intracellular stability and conservation of circRNAs. CircRNAs play more than one role in cells, and some regulate gene expression by regulating mRNA expression of specific genes [8]. Other circRNAs act as inclusions. Other circRNAs may bind transcription factors that are involved in muscle development or viral transcription. Similarly, circRNAs have different mechanisms involved in the development and progression of cancer [18]. Firstly, it has been reported that a genomic translocation leads to the production of a new circRNA that facilitates cell transformation, stimulates cell activity, and promotes tumor development and progression [19]. Secondly, the downregulation of certain circRNA expression levels also affects tumor progression directly or indirectly [8]. It has been found that overexpressed circITCH may regulate the Wnt/attenuated catenin pathway by regulating the activity of miR-7 and miR-214 to inhibit the development of cancer [20]. Finally, a few circRNAs have tumor-promoting effects, and their upregulation may lead to cancer. According to Yang et al., circAmotl1 is highly expressed in cancer tissue samples and related cancer cell lines, which can promote the proliferation of cancer cells [21]. Similarly, circRNA also plays a regulatory role in osteosarcoma. For example, it has been found that circRNA-0008717 may promote the occurrence and development of OS by targeting and competitively inhibiting the regulatory effects of miR-203 [22]. The circRNA circITGA7 studied in this study was found to have differential expression between cancer cells and normal cells. This suggests that circITGA7 may be involved in the development and progression of tumor tissues.

In this study, we mainly discussed the function and mechanism of circITGA7 in OS. Studies have clarified that the expression of circITGA7 in osteosarcoma tissues is significantly lower than that in paracancer tissues. Similarly, the expression level of circITGA7 in the osteosarcoma cell lines is also lower than that of the normal colorectal mucosal epithelial cell line FHC, and its expression level is correlated negatively with OS tumor size, lymph node metastasis, distant metastasis, and overall TNM staging. In vitro experiments showed that circITGA7 could bind to hsa-miR-370-3p to upregulate its target gene NF1 level and then inhibit Ras pathway, further reduce Ras protein level and the phosphorylation level of Erk and Akt, and finally play a role in inhibiting the growth and metastasis of osteosarcoma. Interestingly, previous studies have shown that circITGA7 is significantly downregulated in colorectal cancer (CRC), inhibiting the proliferation and metastasis of CRC cells in a variety of ways [15, 16]. Our results differ from those of the previous studies in which circITGA7 inhibited CRC cells. We found that in vitro knockout of the circITGA7 gene in the cell line inhibited the proliferation of osteosarcoma cells and reduced the ability of osteosarcoma cells to migrate and invade. Some studies show that the function of miR-370 was achieved mainly by regulating the activity of the target miR-370. For example, Yungang et al. found that miR-370 targeted FoxM1 functions as a tumor suppressor in large square cell carcinoma (LSCC) [23]; Zhang et al. showed that miRNA-370 has the tumor suppressive role by targeting FoxM1 in acute myeloid leukemia [24].

MicroRNAs are small noncoding RNAs of less than 30-nucleotide long. However, miRNA plays an extremely important role in the life activities of cells, affecting various physiological and metabolic activities of cells, including proliferation, differentiation, and apoptosis [25]. There is increasing evidence that abnormal upregulation or downregulation of miRNAs is associated with the occurrence and development of a variety of human tumors. For example, miRNA-29c inhibits the ability of lung cancer cells to migrate and invade [26]. Similarly, studies have shown that miR-370 has a potential carcinogenic effect by directly targeting the PDHB gene to promote the development of melanoma [27]. Studies have shown that miR-370 inhibits liver cancer or hepatocellular carcinoma by directly targeting PIM1, and similar results have been found in esophageal squamous cell carcinoma (ESCC) [28]. miR-370 impedes cell proliferation and tumor growth by directly targeting PIM1. PIM1 is a serine/threonine-specific kinase 1 involved in the development of cancer cells [29]. PIM1 is an oncogene that can promote the growth and metastasis of colorectal cancer (CRC). Its expression is positively correlated with the progression of CRC and can predict the prognosis of patients with CRC [30]. PIM1 is significantly overexpressed in gallbladder cancer (GBC) tissue, and its expression level is positively correlated with clinical malignancies and poor prognosis. PIM1 is a promising therapeutic target for the treatment of human GBC [31]. In triple-negative breast cancer (TNBCs) tumors and their cell models, PIM1 expression is related to several transcription signals involving the transcription factor MYC. PIM1 is a malignant-cell-selective target in TNBC, and PIM1 inhibitors have potential use in sensitizing TNBC to chemotherapy-induced apoptotic cell death [32]. Our results show that circITGA7 regulates the activity of miR-370, thereby affecting the activity of PIM1, which promotes the proliferation and metastasis of OS cells.

There are still some limitations in this study. First of all, the number of osteosarcoma tissue samples we used in the study was small. Secondly, the expression pattern and prognostic value of miR-370 and PIM1 should be further explored. Therefore, further research is needed to clarify the potential mechanism of miR-370 and PIM1 in osteosarcoma.

In summary, in this study, we found through a series of experiments that circITGA7 could act as a sponge to competitively inhibit the activity of miR-370 and regulate the physiological activity of osteosarcoma cells through miR-370/PIM1, thus promoting the development of osteosarcoma cells. This provides the possibility of biomarkers for the early screening, diagnosis, and later treatment monitoring of OS.

## Figures and Tables

**Figure 1:** Expression and influence of circITGA7 in OS. (a) The expression of circITGA7 in 15 pairs of OS tissues and corresponding normal tissues. (b) The relative expression of circITGA7 in four OS cell lines (MG-63, HOS, U2OS, and SW1353) and one normal cell line (hFOB 1.19). (c) The relative expression of circITGA7 in cells after circITGA7 knockdown. (d, e) Relative OD 450 value of U2OS and SW1353 with si-circ or si-con. ^∗^*P* < 0.05, ^∗∗^*P* < 0.01.

**Figure 2:** Cell migration and invasion by transwell assay. (a, b) Number of migrations in SW1353 and U2OS cells after different treatments. (c, d) The relative invaded numbers of SW1353 and U2OS cells with si-circITGA7 were less. ^∗^*P* < 0.05, ^∗∗^*P* < 0.01, and ^∗∗∗^*P* < 0.001.

**Figure 3:** miR-370 is the target of circITGA7. (a, b) The relative luciferase activity in SW1353 and U2OS cells cotransfected with miR-370 and circ wt or miR-370 and circ mut. (c) After knocking down circITGA7, the miR-370 expression in OS cells. (d) The relative luciferase activity of PIM1 wt but not PIM1 mut was reduced by miR-370. (e) miR-370 overexpression lowered the PIM1 mRNA expression, while anti-miR-370 increased the PIM1 mRNA expression. (f) Anti-miR-370 compensated for the decreased PIM1 mRNA expression caused by si-circITGA7. ^∗^*P* < 0.05, ^∗∗^*P* < 0.01, and ^∗∗∗^*P* < 0.001.

**Figure 4:** miR-370 reversed the effect of circITGA7 and the effect of PIM1 on OS cells. (a) Overexpression of miR-370 in U2OS cells decreased OD 450 value. (b) OD 450 value was higher in SW1353 cells with anti-miR-370. (c) Relative migration cells of U2OS overexpressed miR-370. (d) The relative migration of SW1353 cells with low miR-370 expression. (e, f) OD 450 value under the low expression of miR-370 after the OS cells knocked down the circITGA7. (g, h) Migrated cells under the downregulation of miR-370 in OS cells after circITGA7 knockdown. (i) OD 450 value of OS cells with si-PIM1 and anti-miR-370. (j) Relative migrated cells of OS cells with si-PIM1 and anti-miR-370. ^∗^*P* < 0.05, ^∗∗^*P* < 0.01, and ^∗∗∗^*P* < 0.001.

## Data Availability

The data used to support the findings of this study are available from the corresponding author upon request.
